The article "Stem Cells Promote the Regeneration of Knee Joint Degenerative Bone and Articular Cartilage" was retracted in 2022. Reason: concerns about the peer review.

# Stem Cells Promote the Regeneration of Knee Joint Degenerative Bone and Articular Cartilage

**DOI:** 10.1155/2022/9533211

**Published:** 2022-03-24

**Authors:** Min Zheng

**Affiliations:** Orthopaedics, Shanghai Punan Hospital of Pudong New District, Shanghai 200125, China

## Abstract

Cartilage damage has a certain ability to spontaneously repair, but the repaired tissue often shows the phenomenon of cartilage terminal differentiation, which causes irreversible damage to its structure and function and seriously affects the quality of life and work of patients. It is of great significance to study the problems encountered in the process of cartilage damage repair. This article mainly studied stem cells to promote the regeneration of knee joint degenerative bone articular cartilage. First, the animal articular cartilage defect is modeled, 10 ml of animal venous blood is drawn, 0.5 ml of PRP is collected by centrifugation, mixed with cartilage fragments, and transplanted into the defect area into a gel. In the BMSCs group, 1 ml of BMSCs with a cell concentration of 107 cells/ml was injected intra-articularly. The histological chromosomes were observed after 6 weeks and 12 weeks, and the effect of cartilage tissue repair was analyzed and evaluated, and the related data were statistically analyzed. We evaluated the spontaneous repair ability of partial cartilage damage, full-thickness cartilage damage, and osteochondral damage. Furthermore, for partial cartilage damage repair, by using the cartilage damage in vitro model and biomaterials to simulate the in vivo microenvironment, the adhesion and cell morphology on the surface of partial- and full-thickness cartilage damage were evaluated, and the experiments were further used to evaluate the exogenous and internal induced migration effect of source on cultured cells in vitro. In the cell concentration study, the cartilage repair effect increased with the increase in concentration within a certain range, and the tissue repair ability remained stable when the concentration exceeded 107 cells/ml. Using ECM-oriented scaffolds to compound autologous BMSCs, tissue-engineered cartilage was successfully constructed, which had the histological and biochemical characteristics of normal cartilage tissue, and better repaired the damaged articular cartilage of large animals.

## 1. Introduction

Joint degeneration is usually caused by trauma or other pathological causes of cartilage and osteochondral damage, which ultimately leads to the complete destruction of the entire joint structure, resulting in total loss of joint function. Current research shows that although certain biological agents can delay the deterioration of the disease and reduce the pain of patients to varying degrees, these drugs cannot effectively promote tissue regeneration. Due to the extremely limited ability of articular cartilage regeneration, arthroplasty has become an inevitable surgical method to restore joint function in the late stage. This review describes the clinical repair techniques widely used to repair defects in articular cartilage and discusses the long-term and short-term clinical effects of these techniques. At the same time, in the next 10 years, the combination of therapeutic methods and the development of regenerative biologics is expected to cure joint cartilage damage and restore joint function. These products include cell-based and cell-free materials, such as autologous and allogeneic cells, and a variety of versatile cell-based technologies. The key to these technologies is to use tissue engineering methods to transform biotechnology into clinical products, thus playing an important role in these aspects.

The article "Stem Cells Promote the Regeneration of Knee Joint Degenerative Bone and Articular Cartilage" was retracted in 2022. Reason: concerns about the peer review.

Articular cartilage injuries are very widespread, such as trauma, genetics, and degenerative changes. In the process of postinjury repair, what factors are at work? A large number of experimental studies have proved that there are indeed some proteins in the process of articular cartilage repair that play an important role in the regulation of cartilage metabolism [1], but these are known single proteins, and there is no analysis and research on all proteins that may play a role in the repair process. Therefore, it is necessary to use stem cells to promote the study of all protein abnormal changes in the joint synovial fluid during the articular cartilage repair process [2]. This review aims to study the role of these stem cells in cartilage repair and provide new ideas and new methods for the clinical treatment of cartilage damage.

Osteoarthritis (OA) is a rheumatic disease that causes chronic pain and disability. There is no effective treatment. Vonk LA studied the role of extracellular vesicles (EVs) secreted by human bone marrow mesenchymal stem cells (BMMSCs) in the repair of human OA cartilage. He tested and observed the effect of BMMSC-EVs on OA cartilage inflammation; treated TNF-*α*-stimulated OA chondrocyte monolayer culture with BMMSC-EVs; 48h later, used qRT-PCR to detect proinflammatory gene-expressing chondrocytes; and 4 weeks later, 1, 9-dimethylmethylene blue (DMMB) analyzed its glycosaminoglycan content. In addition, paraffin sections of the regenerated tissue were stained for proteoglycan (saffron-O) and type II collagen (immunostaining). His method proved that BMMSC-EVs are an important medium for cartilage repair, but the detailed principle is still not proven [3].

The article "Stem Cells Promote the Regeneration of Knee Joint Degenerative Bone and Articular Cartilage" was retracted in 2022. Reason: concerns about the peer review.

Cartilage tissue engineering is an optimized combination of a new type of scaffold, cell source, and growth factors and has become a promising strategy for cartilage regeneration and repair. Fu N. studied the role of polycaprolactone-polyethylene glycol-polycaprolactone (PCL-PEG-PCL) PCEC scaffold in cartilage repair. He first prepared PCEC thin films and tested their properties using scanning electron microscopy and atomic force microscopy. After cell inoculation, the morphology of cells on the PCEC membrane (SCC rat adipose-derived stem cells and muscs green fluorescent mouse adipose stem cells) was observed by scanning electron microscopy and fluorescence microscopy. The Ccts-8 method was used to detect cell viability on PCEC membranes. In addition, complete cartilage defects were created in rats, and the PCEC film was embedded to evaluate its healing effect for 8 weeks. His method is one-sided and does not objectively explain the results of the experiment [4]. Bone marrow mesenchymal stem cell (MSC) therapy is currently under clinical trial for the treatment of cartilage injury. Although cell therapy shows therapeutic effects, there are still logistic and operational challenges associated with transport restrictions, storage, and proper handling. Exosomes are double lipid membrane vesicles secreted by nanoscale cells that exist in the MSC secretion body. They have been found to mediate the regeneration and immune regulation functions of MSCs in animal models. Zhang S hypothesized that human MSC exosomes may represent a new cell therapy method to promote cartilage regeneration. Therefore, they purified exosomes from the conditioned medium of human embryonic mesenchymal stem cells and evaluated their ability to repair critical size osteochondral defects in an immunocompetent rat model. His method is based on the assumption of no actual situation, and the credibility is not high [5].

This study tested the effects of BMSC-Exos and articular chondrocyte-derived exosomes (AC-Exos) on cartilage regeneration through a series of experiments. PIC hydrogel is used as a biological carrier, loaded with BMSC-Exos and AC-Exos, and the repair of sheep's articular cartilage defects is used as an animal model. The in vivo experiment was evaluated by gross ICRS, cartilage repair score, histological staining, and immunohistochemical staining. The effect of different exosomes in repairing cartilage damage and the degree of fibrosis of new tissues were observed; in vitro experiments were conducted to coculture BMSC-Exos and AC-Exos with chondrocytes and observed using a light microscope, western blot, flow cytometry, and immunofluorescence technology to detect changes in the phenotype of chondrocytes.

The article "Stem Cells Promote the Regeneration of Knee Joint Degenerative Bone and Articular Cartilage" was retracted in 2022. Reason: concerns about the peer review.

## 2. Osteoarticular Cartilage Regeneration

### 2.1. Impact of Degenerative Knee Joint Pain

There are four main aspects that affect the quality of life of the elderly, including physical health, mental health, and external economic and social activities. The most important thing for the elderly is physical health. Since birth, old age, sickness, and death are the normal natural aging processes of people; when there is a disease, it will directly affect the health of the elderly. Because it is not healthy enough, their natural aging process will naturally accelerate, which is directly reflected in the gradual degradation of various body functions, so that the physical and mental health of the elderly suffer a double blow. Degenerative musculoskeletal disease and other diseases have a high incidence in the elderly [6].

The structure of the knee joint is more complex, with the upper femur and the lower tibial plateau, as well as the overlying ligament muscle tissue, so the degenerative changes of the muscles around the knee joint will cause corresponding changes in the knee joint structure. Studies have shown that people lose 1% to 3% of their muscle strength every day without exercise [7]. In elderly people over the age of 65 years, because they have retired and rarely take part in physical activity, this will exacerbate the changes brought about by this degenerative muscle loss. With the improvement of living standards and the development of intelligence, a mobile phone can complete all things in basic life, and people's laziness will also increase accordingly. If you do not exercise or exercise every day, the muscles and joints will not be able to meet people's needs for exercise, which will cause the ligaments around the knee joint to become abnormally stressed, the knee joint will become unstable, and even walking and legs will become unstable. As a result, the force line structure of the knee joint will be changed. The change of the knee joint force line will cause the two joints of the knee and the upper and lower joints to move out of the groove. The movement out of the groove will excessively grind the ligaments around the knee joint and cause pain [8]. The imbalance of muscle strength can also cause the relative position of the two bones of the knee joint to move back and forth and left and right, and this movement exacerbates the occurrence of knee pain.

Degenerative knee pain has become a common phenomenon. Degenerative knee pain is a major factor affecting the quality of life of the elderly. It often manifests as pain when going up and down stairs, walking, unstable and bumpy, and poor flexion and extension. In severe cases, loss of joint function may occur, leading to loss of labor and living ability [9, 10]. There are about 250 million patients with knee pain around the world, and the elderly account for 30% of those with knee pain. There are about 210,000 elderly patients in China who undergo knee replacement surgery. According to relevant statistics, the number of knee pain patients over the age of 60 years in my country can reach one-half, and the disability rate can reach five-eighths. Knee pain in the elderly has attracted increasing attention from the society. How to change this situation has brought us a lot of thinking [11].

The article "Stem Cells Promote the Regeneration of Knee Joint Degenerative Bone and Articular Cartilage" was retracted in 2022. Reason: concerns about the peer review.

### 2.2. Cartilage Tissue Engineering

According to the composition of the matrix, cartilage can be divided into elastic cartilage, fibrocartilage, and hyaline cartilage. Articular cartilage is hyaline cartilage tissue that grows on the surface of the joint. Hyaline articular cartilage is an avascular and nerveless tissue composed of chondrocytes, water, collagen fibers, and proteoglycans [12].

The emergence of tissue engineering technology has brought another possibility for the repair and reconstruction of organs and tissues [13]. Cartilage tissue engineering is to plant in vitro chondrocytes or stem cells with differentiation ability into a biocompatible three-dimensional scaffold. The scaffold can simulate natural cartilage in structure and function and can interact with the surrounding cartilage after being implanted into the cartilage defect. The tissues are well fused to repair and regenerate cartilage tissue and can maintain the function of new cartilage for a long time without cartilage degradation and finally realize the purpose of repairing cartilage defects caused by trauma, congenital malformations, and diseases [14, 15].

Cartilage tissue engineering includes cartilage seed cells, scaffolds, and sensor signals. Cells from various sources have been used as seed cells for cartilage tissue engineering, such as chondrocytes, fibroblasts, and stem cells. Regulatory signals such as growth factors have the effect of accelerating and promoting cartilage repair. Growth factors can be added to the culture medium to promote cell growth and differentiation when cells are cultured in vitro, and growth factors can also be loaded into the scaffold to promote cell differentiation and organization of regeneration. Many growth factors, such as TGF-*β*, PDGF-BB, FGF, BMP, and IGF, have been used in cartilage tissue engineering [16].

Although the method of tissue engineering has been successful in the regeneration of many soft tissues, there are still many unsolved problems in cartilage tissue engineering. On the one hand, the structure and properties of the cartilage itself make it difficult to repair itself after injury. On the other hand, how to find a more advanced, more convenient, and more controllable three-dimensional scaffold preparation technology is particularly important. The prepared tissue-engineered cartilage scaffold can simulate the internal structure and physiological composition of natural cartilage, to give cells and tissues the best growth microenvironment. There are still challenges to achieve the ideal functional replacement.

The article "Stem Cells Promote the Regeneration of Knee Joint Degenerative Bone and Articular Cartilage" was retracted in 2022. Reason: concerns about the peer review.

### 2.3. Cartilage Regeneration Method

Among the various types of stem cells in the human body, stem cells extracted from the bone marrow have many unique advantages in clinical applications. Due to their relatively easy separation and strong reproductive capacity, it is convenient for us to obtain them from donors and store them in readymade cell banks. In addition, clinical experiments have confirmed that a large number of clinical experiments conducted in vitro and in vivo have found that human bone marrow mesenchymal stem cells can differentiate into cartilage tissue and bone tissue and play an important role in the regeneration of osteochondral defects and cartilage defects [17]. Specifically, bone marrow mesenchymal stem cells are derived from patients with osteoarthritis, and they have shown in vitro that they can produce proteoglycans, type II collagen, and TGF − *β*_1_ that maintain the shape of chondrocytes in a three-dimensional scaffold. Another notable feature is their ability to selectively migrate to diseased tissues and organs. They are found to secrete cytokines that inhibit cell proliferation in cartilage defects. These cytokines are thought to play an essential role in allograft and xenotransplantation. In the context of cartilage repair, MSCs can activate specific tissue repair systems that can be used to nourish cartilage and promote its growth and repair by directly releasing synthetic, proliferative, and regenerative factors into cartilage damage. Through the release of chemokines to create a regenerative environment, bone marrow mesenchymal stem cells may also drive endogenous stem cells into the cartilage-damaged area to repair damaged cartilage tissue [18].

At present, most studies on cartilage regeneration through stem cells are bone marrow-derived mesenchymal stem cells. Although the extraction process of the bone marrow is very painful, it is an effective method to obtain stem cells. However, stem cells can also be obtained from other sources, including adipose tissue, muscle, cortical cancellous bone, synovium, periosteum, and umbilical cord. Human adipose stem cells are the easiest to obtain. In vitro studies have shown that these stem cells have proliferation and differentiation capabilities similar to bone marrow mesenchymal stem cells. Adipose-derived stem cells are considered an ideal source of stem cells due to their relatively strong in vitro isolation ability, anti-inflammatory properties, and no immunogenicity. Compared with stem cells from other sources, their proliferation and differentiation abilities are unlikely to be affected by individuals. The effect of age: by injecting adipose stem cells into the knee joints of elderly patients suffering from knee arthritis, combined with arthroscopic minimally invasive surgery for joint cavity lavage, the clinical feasibility and safety of human adipose stem cells in the treatment of degenerative cartilage diseases have been studied. The result of the treatment is to improve body function and promote articular cartilage repair, thereby alleviating the pain of the patient's knee joint [19]. However, similar to the combined injection of bone marrow mesenchymal stem cells, this technology also has some similar problems. These problems include the number of cells required to promote cartilage regeneration, whether one injection or more injections are required to achieve the desired effect, the best time window for injection, and the long-term safety of this technology. In addition, some evidence of further improvement needs to be provided by tissue biopsy MRI.

The article "Stem Cells Promote the Regeneration of Knee Joint Degenerative Bone and Articular Cartilage" was retracted in 2022. Reason: concerns about the peer review.

## 3. Experimental Study on Regeneration of Osteoarticular Cartilage

### 3.1. Research Object

The oriented scaffold facilitates the adhesion and growth of seed cells in the scaffold, facilitates the uniform distribution of seed cells inside the scaffold, and helps the seed cells arrange in the scaffold into the arrangement of cells in natural articular cartilage. This determines the structure and functional characteristics of the new organization. This is of great significance for the construction of functional tissue-engineered cartilage. In previous studies, the oriented scaffold combined with autologous bone marrow stem cells can better repair rabbit knee joints after cartilage orientation, but there is no report on its use in repairing articular cartilage defects in large animals.

Bone marrow stromal stem cells have multidirectional differentiation potential and convenient sources. Cells derived from autologous sources have no effect on the body's donor area. They can proliferate rapidly in vitro and will not lose their stem cell characteristics after multiple passages. They are currently available in cartilage tissue engineering, one of the sources of seed cells of concern. However, the previous research work was based on the chondrogenic induction of small animal bone marrow stem cells, and the long-term effect of the induction has not been evaluated for safety. Therefore, this study selected autologous bone marrow stromal stem cells as seed cells and repaired sheep's articular cartilage defects without any inducing factors after the composite orientation scaffold.

The article "Stem Cells Promote the Regeneration of Knee Joint Degenerative Bone and Articular Cartilage" was retracted in 2022. Reason: concerns about the peer review.

### 3.2. Cell Culture and Construction of Tissue Engineered Cartilage Tissue

The obtained cartilage tissue was send to the clinical cell culture room for cultivation. In strict accordance with the requirements and standards of the China Pharmaceutical and Biological Products Inspection Institute, the autologous chondrocytes are separated, cultured, expanded, and quality monitored. The cultivation period is 14–21 days. The isolated primary cells were expanded to 107 at low density. Seed cells were in vitro. Composite three-dimensional scaffold and the operation follows the standardized operation process of tissue-engineered cartilage transplantation.

They were cultured in vitro for a total of 2-3 weeks, a second small incision transplantation operation was performed, and the constructed tissue-engineered cartilage tissue was implanted back into the defect site. The operation followed the standard operating procedure of tissue-engineered cartilage transplantation. On the day of surgery, the tissue-engineered cartilage tissue is transferred to the hospital, the cell biochemical function is tested at the same time, and the culture solution is tested for bacteria and mycoplasma to ensure the quality of the implanted tissue and is free from contamination. Surgical method: Make a small incision to cut the joints, use a sharp blade to cut vertically around the damaged cartilage to the subchondral bone, and use a circular curette to debride the damaged subchondral bone tissue. Trim the tissue to be transplanted into a defect shape, and fix the tissue-engineered cartilage tissue on the edge of the defect with a 6–0 threaded needle absorbable suture (with the periosteal germinal layer facing the cartilage surface). Seal the suture area with fibrin glue. Finally, check the graft fixation, passively extend and flex the joint several times, and suture the wound after confirming that there is no displacement.

### 3.3. Mechanical Test

The mechanical test is used to evaluate the compression performance of the repaired tissue. First, the sample is fixed to the base of the mechanical tester (model 5543, Instron, Canton, MA), and the position is adjusted so that the center of the defect is directly below the compression mold. The compression test is performed with a force of 10N. The speed is set at 0.06 mm/min. When the cartilage layer is compressed to 20% of the thickness of the cartilage layer, the compression is stopped and the compression is allowed to return to the original position. The slope of the stress-strain curve at this time is the measured compressive modulus (MPa). Before the mechanical test, the frozen samples are placed in PBS at room temperature for 3-4 hours to fully equilibrate.

The article "Stem Cells Promote the Regeneration of Knee Joint Degenerative Bone and Articular Cartilage" was retracted in 2022. Reason: concerns about the peer review.

### 3.4. Testing Indicators

Observe the general shape, color, texture, and volume changes of the cell-material complex after one week. Observe the survival and distribution of cells in the cell-material complex after one week of culture. Take the cell scaffold complex that has been cultured for one week, rinse with PBS, and immediately freeze the sections. The sections will be air-dried and fixed with 95% alcohol for AO-PI staining and Hoechst 33258 fluorescent staining; observe the bone marrow stem cells on the scaffold under an inverted microscope.

## 4. Analysis of Osteoarticular Cartilage Regeneration

### 4.1. Analysis of the Influence of BMSC-Exos and AC-Exos on the Maintenance of the Normal Phenotype of Chondrocytes

We stained the envelopes of BMSC-Exos and AC-Exos with green and red fluorescence with membrane fluorescent dyes and cocultured them with chondrocytes. Through fluorescence microscopy, we found that a large number of green and red fluorescences were accumulated in the cytoplasm of chondrocytes. It is suggested that both exosomes can be taken up by chondrocytes in large quantities, and the two exosomes can enter chondrocytes to play a role [20].

When chondrocytes are cultured in vitro, they will gradually dedifferentiate as the number of culture passages increases, losing the unique phenotype of chondrocytes. The tissue obtained by expansion of such dedifferentiated chondrocytes is usually fibrocartilage [21]. The normal articular cartilage in the body is hyaline cartilage tissue, which is composed of mature cartilage cells with a good phenotype and the extracellular matrix secreted by them [22]. Therefore, in the process of cartilage cell expansion, how to effectively maintain the phenotype of cartilage cells has become an important factor in the success of cartilage repair. In this experiment, BMSC-Exos and AC-Exos were cocultured with chondrocytes to detect whether these two exosomes affect the maintenance of the chondrocyte phenotype. Western blot results showed that the expression of the specific marker Sox9 of chondrocytes treated with BMSC-Exos gradually decreased from the 4th to the 10th passage of cell culture, while for the chondrocytes treated with AC-Exos, Sox9 always maintained high expression but no expression decrease.

The article "Stem Cells Promote the Regeneration of Knee Joint Degenerative Bone and Articular Cartilage" was retracted in 2022. Reason: concerns about the peer review.

As shown in Figure 1, the results of flow cytometry showed that when chondrocytes were cocultured with BMSC-Exos at OR in the 10th passage, the percentages of Sox9 and Aggrecan-positive expression cells were 3.3 ± 0.69% and 2.8 ± 0.53%, respectively, while for chondrocytes after AC-Exos treatment, the positive expression rates of Sox9 and Aggrecan in the 10th passage cells reached 92.3 ± 0.68% and 94.1 ± 0.46%, respectively. Light microscopy results showed that the cell morphology of chondrocytes treated with BMSC-Exos gradually changed from oval to elongated spindle shape, suggesting that BMSC-Exos did not change the dedifferentiation trend of cells. The chondrocytes treated with AC-Exos always maintain an oval cell shape [23].

The results of immunofluorescence staining showed that the expression of Aggrecan (red fluorescence) of chondrocytes treated with BMSC-Exos was significantly reduced from the 4th generation, while for chondrocytes treated with AC-Exos, the expression of Aggrecan always remained at a higher level.

### 4.2. Detection of Intracellular Iron in Magnetically Labeled BMSCs by Atomic Absorption Spectrometer

As shown in Table 1, the absorption of superparamagnetic iron oxide correlates with the SPIO concentration. The intracellular iron increased with the increase of the labeling concentration, reaching a peak at 8 *μ*g/ml, and the average cellular iron content was 2.77 ± 0.93 mmol/L. When SPIO continued to increase, the intracellular iron showed a downward trend [24]. Through this result, we can find that too high concentrations of SPIO markers (10 *μ*g/ml and 12 *μ*g/ml) will reduce the uptake of SPIO by cells.

As shown in Table 2 and Figure 2, in the past, SPIO coated with dextran has a short in vivo degradation time, which is difficult to meet the time requirements of tissue engineering tracing, and because its surface is negatively charged, it is not easy to be taken up by cells, so transfection is required. This experiment uses self-synthesized PEI to modify SPIO particles to prepare a new type of SPIO with a positive charge on the surface. When the final concentration of iron content is 8 *μ*g/ml or more and the cells are cocultured for 24 hours, the positive rate is found by the microscope after staining with Prussian blue. Up to 99%, it proves that the new SPIO has been successfully transferred into BMSCs with extremely high labeling efficiency [25]. Experimental research shows that this new type of SPIO can be directly swallowed by cells to label stem cells, without mixing with transfection agents, and is easy to operate. The mechanism is that the surface of mesenchymal stem cells is negatively charged, while the surface of the newly prepared PEI/SPIO is positively charged. It can directly attract each other to OR on OR at the cell surface through positive and negative charges and enter the cell by endocytosis. A mixture of positively charged transfection agents should be used. Studies have shown that the time for SPIO to degrade in vivo and excluded from the body has no correlation with the particle size but is related to the molecular weight of the embedding agent and the hydrophilicity of the surface. PEI has good hydrophilicity, which can be extended by adjusting the molecular weight. The trace time of the labeled cells is closer to the time of cartilage defect repair and healing.

The article "Stem Cells Promote the Regeneration of Knee Joint Degenerative Bone and Articular Cartilage" was retracted in 2022. Reason: concerns about the peer review.

### 4.3. Extraction of hiPS-MSC-Exos and Preparation of EHG Hydrogel

As shown in Figure 3, the nanoparticle analysis results show that the extracted hiPS-MSC-Exos has a particle size range of 50–150 nm; TEM results show that hiPS-MSC-Exos is spherical or elliptical; and western blot detection results show that the above results confirmed the successful extraction of hiPS-MSC-Exos. The rheological test results show that after irradiating the EHG precursor solution with a 395 nm LED light source for 20 seconds, an EHG hydrogel with a stable three-dimensional structure is formed.

As shown in Figure 4, we tested the integration of EHG hydrogel with cartilage and its ability to recruit cells in cartilage defects through in vivo experiments. Scanning electron microscopy results showed that the EHG hydrogel and cartilage tissue were tightly connected, and no gaps were found between the interfaces, suggesting that EHG formed a tight integration with cartilage through chemical cross-linking. The results of HE staining showed that the EHG hydrogel was completely and tightly attached to the surrounding cartilage tissue at the osteochondral defect, and the EHG hydrogel was tightly integrated with the subchondral bone at the base of the defect. The tight integration of the osteochondral tissue allows the exosomes in the EHG hydrogel to directly contact the cells in the surrounding tissues, which can regulate the surrounding cells.

We further studied the regulation effect of EHG hydrogel on the cells surrounding the defect through in vivo experiments. The results of DAPI staining showed that the number of cells in the defect in the EHG group was significantly higher than that in the HG group. The results of HE staining showed that chondrocytes, BMSCs, and inflammatory cells were seen in the defect. This result suggests that EHG hydrogels can efficiently recruit chondrocytes and BSMCs around the defect into the defect site.

## 5. Conclusions

Cartilage tissue cannot heal by itself after injury, and autologous chondrocyte transplantation is limited by the lack of cell source and quantity. From the perspective of tissue-specific stem cells, this study confirmed that cartilage tissue has stem cell characteristics and high cell proliferation efficiency regardless of physiological and pathological conditions. The appearance of such cells may be due to changes in the environment, and related surface markers are dynamically changing.

The article "Stem Cells Promote the Regeneration of Knee Joint Degenerative Bone and Articular Cartilage" was retracted in 2022. Reason: concerns about the peer review.

Experiments in this article confirm that hiPS-MSC-Exos can effectively repair cartilage damage and promote hyaline cartilage regeneration. The results of in vitro experiments confirmed that hiPS-MSC-Exos can significantly enhance the proliferation and migration of chondrocytes and BMSCs. This result suggests that hiPS-MSC-Exos has the function of significantly promoting cartilage cell regeneration and repairing cartilage damage, showing a broad transformation application prospect.

Part of the cartilage is damaged, and its matrix microenvironment is not easy for cells to adhere to and lacks small biological molecules that can effectively induce cell migration. Therefore, we use biomembrane materials combined with matrix cell-derived factors to construct bioactive materials to promote and adhere to migration and then open cartilage repair spontaneously; in osteochondral damage, there are a large number of bone marrow-derived seed cells in the matrix microenvironment to participate in the repair, but in the environment of osteochondral damage, the bone system is more inclined to differentiate, resulting in abnormal cartilage terminal differentiation. Therefore, we used collagen fragrant silk double-layer scaffolds combined with parathyroid hormone-related proteins to inhibit the terminal differentiation of cartilage, promote the process of cartilage formation, and improve the quality of spontaneous cartilage repair.

## Figures and Tables

**Figure 1:** The effect of chondrocyte phenotype maintenance.

**Figure 2:** SI values of SPIO labeling sequences at different concentrations.

**Figure 3:** Particle size range.

**Figure 4:** Preparation of EHG hydrogel.

**Table 1:** Intracellular element content statistics after 24 h incubation.

Labeling concentration (ug/ml)	4	6	8	10	12
Intracellular iron content (mmol/L)	0.79	1.24	2.76	2.34	2.23

**Table 2:** SI values of MRI ^*∗*^ SET2WI sequence of SPIO labeled BMSCs at different concentrations.

Concentration (*μ*g/ml)	1	2	3	4	5	6	7
4	641.45	609.81	490.23	439.99	359.09	308.99	227.55
6	675.67	563.91	528.75	432.99	363.19	307.49	235.66
8	637.62	582.13	530.87	460.00	357.28	287.25	230.09
10	656.92	608.09	494.22	465.53	393.46	311.10	222.00
12	671.29	565.33	533.43	441.57	356.80	322.65	213.80

The article "Stem Cells Promote the Regeneration of Knee Joint Degenerative Bone and Articular Cartilage" was retracted in 2022. Reason: concerns about the peer review.

## Data Availability

This article does not cover data research. No data were used to support this study.

## References

[1] Prabhakar A., Lynch A. P., Ahearne M. (2016). Self-assembled infrapatellar fat-pad progenitor cells on a poly-*ε*-caprolactone film for cartilage regeneration. *Artificial Organs*.

[2] Chen X., Zhang R., Zhang Q. (2019). Chondrocyte sheet in vivo cartilage regeneration technique using miR-193b-3p to target MMP16. *Aging*.

[3] Vonk L. A., van Dooremalen S. F. J., Liv N. (2018). Mesenchymal stromal/stem cell-derived extracellular vesicles promote human cartilage regeneration in vitro. *Theranostics*.

[4] Fu N., Liao J., Lin S. (2016). PCL-PEG-PCL film promotes cartilage regeneration in vivo. *Cell Proliferation*.

[5] Zhang S., Chu W., Lai R. (2016). Human mesenchymal stem cell-derived exosomes promote orderly cartilage regeneration in an immunocompetent rat osteochondral defect model. *Cytotherapy*.

[6] Zhang S., Hamid M. R., Wang T. (2020). RSK-3 promotes cartilage regeneration via interacting with rpS6 in cartilage stem/progenitor cells. *Theranostics*.

[7] Yusoff B. M., Ramlan M., Chin S. (2019). Arthroscopic evidence of cartilage regeneration in severe knee cartilage defects and osteoarthritis following treatment with allogeneic umbilical cord-derived mesenchymal stromal cells (Chondrocell-Ex). *Cytotherapy*.

[8] Verdoni F., Compagnone D., Grasso F. (2019). Chemical and physical influences in bone and cartilage regeneration: a review of literature. *Journal of Biological Regulators and Homeostatic Agents*.

[9] Zhang S., Hu P., Liu T. (2019). Kartogenin hydrolysis product 4-aminobiphenyl distributes to cartilage and mediates cartilage regeneration. *Theranostics*.

[10] Cassani S., Olson S. D. (2020). A hybrid model of cartilage regeneration capturing the interactions between cellular dynamics and porosity. *Bulletin of Mathematical Biology*.

[11] Szychlinska M. A., D’Amora U., Ravalli S., Ambrosio L., Di Rosa M., Musumeci G. (2019). Functional biomolecule delivery systems and bioengineering in cartilage regeneration. *Current Pharmaceutical Biotechnology*.

[12] Santanna J., Fernandez T. L., Bueno D. F., Pinheiro C. C., Hernandez A. J. (2020). Cartilage regeneration with human dental pulp stem cells - a systematic review. *Cytotherapy*.

[13] Johnstone B., Stoddart M. J., Im G. I. (2020). Multi disciplinary approaches for cell based cartilage regeneration. *Journal of Orthopaedic Research*.

[14] Sheykhhasan M., Ghiasi M. S. (2018). Advances in adipose-derived stem cells and cartilage regeneration: review article. *Tehran University Medical Journal*.

[15] Park J. H., Jeon H. Y., Jeon Y. S. (2018). Effect of cartilage regeneration on gellan gum and silk fibroin. *Polymer Korea*.

The article "Stem Cells Promote the Regeneration of Knee Joint Degenerative Bone and Articular Cartilage" was retracted in 2022. Reason: concerns about the peer review.

[16] Landgraeber S., Jäger M., Fickert S. (2017). Knorpelregenerative eh. *Orthopäde, Der*.

[17] Li H., Li M., Yan X. (2017). Nanophase polyaiticglycolic acid/hydroxyapatite composite and mesenchymal stem cells in rat cartilage regeneration. *Journal of Biomaterials and Tissue Engineering*.

[18] Deng C., Yao Q., Feng C. (2017). 3D printing of bilineage constructive biomaterials for bone and cartilage regeneration. *Advanced Functional Materials*.

[19] Piombo V. (2017). Small animal models to understand pathogenesis of osteoarthritis and use of stem cell in cartilage regeneration. *Cell Biochemistry and Function*.

[20] Zhang Q. S., Kurpad D. S., Mahoney M. G., Steinbeck M. J., Freeman T. A. (2017). Inhibition of apoptosis signal-regulating kinase 1 alters the wound epidermis and enhances auricular cartilage regeneration. *PLoS ONE*.

[21] Mc Donald C. K., Moriarty P., Varzgalis M., Murphy C. (2017). The top 50 most cited articles in cartilage regeneration. *BioResearch Open Access*.

[22] Wang L., Huang C., Li Q., Liu L., Luo S., Xiao J. (2018). Adult stem cells and hydrogels for cartilage regeneration. *Current Stem Cell Research and Therapy*.

[23] Choi W. H., Kim H. R., Lee S. J. (2016). Fetal cartilage-derived cells have stem cell properties and are a highly potent cell source for cartilage regeneration. *Cell Transplantation*.

[24] Chen Z., Yan C., Yan S. (2018). Non-invasive monitoring of in vivo hydrogel degradation and cartilage regeneration by multiparametric MR imaging. *Theranostics*.

[25] Shi D., Xu X., Ye Y. (2016). Photo-cross-linked scaffold with kartogenin-encapsulated nanoparticles for cartilage regeneration. *ACS Nano*.

